The article "Study on the Diagnostic Value of Contrast-Enhanced Ultrasound and Magnetic Resonance Imaging in Prostate Cancer" was published in 2022. Journal: Evid Based Complement Alternat Med.

# Study on the Diagnostic Value of Contrast-Enhanced Ultrasound and Magnetic Resonance Imaging in Prostate Cancer

**DOI:** 10.1155/2022/7983530

**Published:** 2022-08-08

**Authors:** Xinnian Pang, Jianhua Zhang, Lvcou Chen, Yang Yuan, Dong Xu

**Affiliations:** ^1^Department of Ultrasound, Tiantai People's Hospital of Zhejiang Province, Taizhou 317500, Zhejiang, China; ^2^Department of Urology, Tiantai People's Hospital of Zhejiang Province, Taizhou 317500, Zhejiang, China; ^3^Department of Ultrasound, Zhejiang Cancer Hospital, Hangzhou 310022, Zhejiang, China

## Abstract

**Objective:**

The aim is to study the different roles of single and joint application of magnetic resonance imaging (MRI) and contrast-enhanced ultrasound (CEUS) in prostate malignant tumors.

**Methods:**

72 patients with prostate masses who underwent CEUS and MRI examination in our hospital from October 2021 and March 2022 were enrolled in this research. The differentially diagnostic roles of CEUS, MRI, and CEUS combined MRI for prostate cancer was assessed on basis of pathological findings as the reference standard. The specificity and sensitivity of the joint application for prostate malignant tumors with various prostate-specific antigen (PSA) levels were also evaluated.

**Results:**

The sensitivity of CEUS, MRI, and the joint application for prostate cancer were 72.1%, 74.4%, and 90.7%, respectively. Compared with single application, the sensitivity of CEUS combined with MRI was significantly higher. The specificity of MRI, CEUS, and the combination of the two for prostate cancer were 82.8%, 79.3%, and 89.7%, respectively, and the statistical differences for specificity were not found. The area under ROC curve (AUC) of CEUS combined with MRI in prostate malignant tumor diagnosis was obviously more than that of CEUS and MRI (*P* < 0.05). CEUS combined with MRI has relative high sensitivity in these patients with different levels of PSA.

**Conclusions:**

Contrast-enhanced ultrasound combined with MRI can significantly improve the sensitivity and specificity of prostate cancer diagnosis so that patients can be better diagnosed in advance.

## 1. Introduction

In western countries, prostate malignant tumor is considered as the common cancer, especially in elderly men [1]. It was reported that the occurrence rate of prostate malignant tumor raised every year, which severely affected the physical and psychological status of these patients [2, 3]. Many studies reported that patients with prostatic cancer in the early phase who underwent timely treatment could gain a more than 5-year survival rate, while those in the end stage showed an obviously less than 5-year survival rate [4]. Early detection of prostate malignant tumor is extremely important for enhancing the quality of life and reducing the death rate. At present, biopsy under the guidance of ultrasound has become the standard method in the diagnosis of prostate malignant tumor. But the shortcomings of technologies are proverbial [5]. Therefore, novel imaging procedures should be recommended as an alternative to characterize and identify the prostate tumors.

Magnetic resonance imaging (MRI) is currently the optimal detection for the findings of prostate malignant tumors. However, using MRI alone has some limitations. It was reported that could MRI only find morphological information and was not able to obtain the internal microstructure of tumor tissues, resulting in difficult evaluation for the risk of prostate tumors [6]. Another study showed that diffusion-weighted MRI could well manifest the tissue of tumor with abundant vascularity; however, the diagnostic role for prostate malignant tumor was debated [7]. In conclusion, MRI has the advantages of thorough research and clear morphological information and can better display tumor tissues with abundant blood vessels. In recent years, contrast-enhanced ultrasonography (CEUS) appeared with the development of advanced techniques in the ultrasound imaging. The value of CEUS in oncologic diagnosis attracts increasing emphasis due to the measurement of moving blood [8]. It was reported that improved cancer identification at CEUS was associated with the better examination of small blood flow in tumors [9]. So far, few data are found regarding the value of MRI plus CEUS for the prostate malignant tumor diagnosis. In this context, this research was performed to study the roles of MRI plus CEUS for prostate tumors and it will provide important evidences for assessing prostate malignant tumor.

## 2. Material and Methods

### 2.1. Basic Data

From October 2021 and March 2022, 72 patients with prostate masses were included in this research; hospital ethics committee approved this trial.

The signed informed consent was provided. The inclusion criteria were as follows: (1) those who were diagnosed as suspicious prostate cancer with over 30 years of age and elevated levels of prostate-specific antigen (PSA) (≥4.0 ng/mL). (2) Those who had no history of radiotherapy, chemotherapy, and endocrine treatment. (3) The examinations of contrast-enhanced ultrasonography, MRI, and prostate biopsy were performed. (4) Complete medical records were obtained and patients were able to cooperate in the research. The exclusion criteria were as follows: (1) History of malignant tumor. (2) History of prostate operation. (3) Hypersensitivity reaction of the contrast agent. (4) Accompaniment with disorders of the blood and immune system, prostatitis, and acute urinary tract infections. (5) Severe renal and hepatic insufficiency, cardio- and cerebrovascular disease, and mental disorders. All the patients were informed about the necessity for pathological detection and about the examination of contrast-enhanced ultrasonography and MRI conducted prior to the biopsy.

### 2.2. Contrast-Enhanced Ultrasonography Examination

Patients were maintained at a left lateral position. The transrectal conventional ultrasound was performed for each patient by LOGIQ E9 type ultrasound equipment (GE Company, USA). All the examination was conducted by two senior doctors who were blinded to this study. Then, the system of ultrasound was switched into the model of contrast-enhanced ultrasonography when the conventional ultrasound was finished. The contrast medium SonoVue (Bracco Suisse SA, Swiss) was injected into the peripheral vein of patients. Next, 5 ml normal saline was injected. The transducer was fixed over the suspicious lesions and regions of interest. The video was real-time dynamically observed for 3 min. Through reviewing the images, the prostate cancer was diagnosed according to the parameters reported by previous studies [10].

### 2.3. MRI Detection

The subjects were kept in the supine position with a proper distended bladder under the condition of steady breaths. The MRI examination was conducted using a 1.5 T Signa HDxt magnetic resonance scanner (GE Company, USA). The scanning scope involved in the whole prostate. T2WI sequence examination was used for analyzing the tumor of the prostate. T2 weighted fat saturation (T2WFS) scans were performed based on the following arguments: TE 100 ms, TR 5500 ms, FOV 230 mm × 230 mm, matrix 320 × 320, slice thickness 4.0 mm. Diffusion-weighted imaging (DWI) was conducted using spin echo-echo planar imaging. The parameters were as follows: *b* values were set as 0 s/mm^2^, 500 s/mm^2^, 1500 s/mm^2^, 2000 s/mm^2^, TR 4000 ms, TE 86 ms, Matrix 180 × 180, FOV 230 mm × 230 mm, slice thickness 4.0 mm. Apparent diffusion coefficient (ADC) imaging was constructed on basis of DWI. The original MRI image was transmitted to Picture Archiving and Communications Systems (PACS) workstation. The corresponding images from MRI were blindly assessed by two experienced radiologists together with prostate imaging report and data system version 2.1 (PI-RADS v2.1). The scoring criteria should refer to the latest version of PI-RADS V2.1 [11]. Three scores or more were considered as prostate cancer. The agreements should be reached by consensus when their views were different.

### 2.4. Prostate Biopsy Examination

After contrast-enhanced ultrasonography and MRI examination, all patients underwent prostate puncture under the guidance of ultrasound, and the standard puncture method was adopted. The puncture specimens from the patients were immediately embedded in paraffin and stained in sections. Two experienced pathologists blindly interpreted the pathological sections. Moreover, prostate cancer was pathologically confirmed by the Gleason scoring system from the International Association of Urological Pathology [12].

### 2.5. Statistical Methods

All the clinical data obtained in the research were analyzed through SPSS version 23.0. The measurement data were shown in the form of mean ± standard deviation. The count data were showed in the form of percentages/cases. The comparison among groups was conducted using *χ*^2^ test. On the basis of the pathological results as the gold standard, the diagnostic value including specificity and sensitivity of CEUS, MRI, and the combined application for prostate cancer was analyzed. Diagnostic efficiency of CEUS, MRI and the combined application for prostatic malignant tumor was also evaluated through receiver operating characteristic (roc). *P* < 0.05 indicated significantly statistical differences.

## 3. Results

### 3.1. General Information

As seen in Table 1, the mean age of patients included in the research was 62.8 ± 6.5 years. The body mass index was 21.5 ± 0.7 kg/m^2^. Disease periods of time were 2.5 ± 0.6 years. The serum PSA level was 69.8 ± 10.4 ng/mL. It showed 23 cases with benign prostatic hyperplasia (BPH), 2 cases with intraepithelial neoplasia, 4 cases with prostatitis, and 43 cases with prostate cancer. Moreover, there were 15 patients with hypertension, 18 patients with diabetes, and 12 patients with hyperlipidemia.

### 3.2. Comparison of Diagnostic Efficiency of CEUS, MRI, and the Combined Application for Prostatic Cancer

The sensitivity of CEUS, MRI, and CEUS combined with MRI for prostate malignant tumor was 72.1%, 74.4%, and 90.7%, respectively. In contrast to CEUS or MRI, the sensitivity of CEUS combined with MRI in prostate cancer was significantly increased (*P* < 0.05). The specificity of CEUS, MRI, and CEUS combined with MRI in prostate malignant tumor was 79.3%, 82.8%, and 89.7%, respectively. The significant differences were not found regarding the specificity for examination of prostate cancer among different methods as shown in Table 2.

### 3.3. Comparison of ROC Results

The AUC of CEUS, MRI, and CEUS combined with MRI for prostate cancer was 0.608, 0.667, and 0.785, respectively. The AUC of CEUS plus MRI diagnosed for prostate cancer was significantly more than that of CEUS or MRI, and there was the obviously statistical difference (*P* < 0.05) as seen in Table 3 and Figure 1.

### 3.4. Diagnostic Efficiency of CEUS Combined with MRI among Different Levels of PSA

When PSA was in the range of 4 ng/mL to 10 ng/mL, the specificity and sensitivity of CEUS combined with MRI for diagnosis of prostate malignant tumor were 78.3% and 100%. When PSA was in the range of 10 ng/mL to 20 ng/mL, the sensitivity and specificity of CEUS combined with MRI for diagnosis of prostate cancer were 81.8% and 60.0%. When PSA was more than 20 ng/mL, the specificity and sensitivity of CEUS combined with MRI in diagnosis of prostate malignant tumor were 66.7% and 100% as seen in Table 4.

## 4. Discussion

In clinical practices, most of patients with early-stage prostate cancer do not have special clinical manifestations. When the clinical symptoms occur, it is usually diagnosed as the advanced stage. The differential diagnosis between prostate cancer and benign tumors was confirmed by the transrectal ultrasound guided biopsies. Many studies showed that the incidences of complications including bleeding and pain make a lot of patients to difficultly agree to the operation of needle biopsy [13]. Thus, the optimal examination technology for prostate malignant tumor is required to be less damage, noninvasive, and less adverse reactions and would be of benefit to a high proportion of patients.

The improvement of diagnostic pathways for prostate cancer is necessary and might be based on the progress of imaging detections. MRI, as a noninvasive examination, has the characteristic of good resolution for soft tissues and could show the invasion of seminal vesicle and extracapsular in prostate malignant tumor. The routine morphological examination of MRI is of great significance for evaluating the tumor size, location and stage, and guiding needle biopsy. This study showed the specificity and sensitivity of MRI for detecting prostate malignant tumor was 82.8% and 74.4%, which was basically similar with the results reported by previous studies [14]. CEUS, as an ultrasound imaging examination, makes an important progress in the diagnosis of malignant tumor. Microvascular imaging during CEUS could clearly display the images of blood flow perfusion and distribution in prostate cancer, which could improve the sensitivity and specificity in the prostate malignant tumor diagnosis. Some trials reported that the increased microvessel density in prostate malignant tumor was correlated with grading of tumors and metastasis and prognosis of patients [15]. In this study, it was showed that the specificity and sensitivity of MRI for detecting prostate malignant tumor were 79.3% and 72.1%. Huang et al. revealed the similar results [16]. However, there were few data regarding the diagnostic efficacy of MRI combined with CEUS in prostate cancer. Aiming at the features of MRI and CEUS, The strong points of both were obtained by the combined application technology. MRI combined with CEUS could not only evaluate the microvessel density in prostate tissues and observe the signal symmetry of the blood flow, but also offer the all-round vision for the physiological anatomy of prostate tissues and show the blood supply in the lesions and its peripheral tissue. The results of this study found that the specificity and sensitivity of CEUS combined with MRI for detecting prostate cancer were 89.7% and 90.7%, which were higher than those in MRI or CEUS. Moreover, the AUC of combined application was significantly higher than that in MRI or CEUS, and the obviously statistical differences were found. It was suggested that MRI combined with CEUS had obvious advantages in the term of prostate malignant tumor diagnosis.

PSA is considered as the commonly clinical indicator in the examination of prostate malignant tumor. PSA was also usually performed as a marker in the screening and assessment of treatment effect in prostate malignant tumor [6]. Previous research studies found that increased PSA levels were closely associated with the clinical phase of prostate malignant tumor and the higher PSA concentration indicated the worse damage of surrounding tissues and malignant degree [17]. This study revealed that MRI combined with CEUS showed a high specificity and sensitivity in patients with different increased PSA concentrations. It also indicated that this combined application technology could limit the number of biopsy cores and enhance the detection of prostate malignant tumor under the biopsy guidance. Some studies reported that the combined application was able to detect the prostate lesions which could not be detected using systematic biopsy [18]. MRI combined with CEUS differentially diagnosed prostate malignant tumor from benign tumors and prostatitis based on various vascular enhancements. This technology strongly allowed features of vascular alterations in the areas of tumor, which was helpful to identify benign inflammatory nodules from neoplastic nodules. The distinguishment of suspected tissues with increased PSA concentration allowed guided biopsy, which would improve the probability of examining a possible malignant tumor.

The current study has several limitations that should be recognized. First, this was a retrospective study, which could not perform blind, randomization, and power calculation. Second, the sample size in this research was not large, which might influence the findings. Third, the clinical data of patients were obtained from single center, which may influence its generalization to other hospitals. In future studies, it was demanded to demonstrate this opinion by expanding the sample size and exploiting multi-center prospective study.

## 5. Conclusions

In summary, although CEUS or MRI revealed relatively high specificity and sensitivity in examining prostate malignant tumor, MRI combined with CEUS yields a higher detective rate of prostate cancer. A satisfactory finding seems to be achieved when the combined application is exploited for patients with different elevated PSA concentrations. If this combined application could be further development, it would be conductive to the prostate cancer monitoring following therapy and to the clearly distinguishment of malignant lesions when focal treatment is conducted. As a future application of CEUS combined with MRI, this technique has the potential to exert an important role in diagnosis and prognosis assessment for prostate cancer and must be further explored. The application of CEUS combined with MRI for diagnosis and treatment would develop a new field in prostate malignant tumor.

## Figures and Tables

**Figure 1:** ROC curve of different examination methods for diagnosis of prostate cancer.

**Table 1:** General data of patients included in the research.

Indicators	Values
Age (years)	62.8 ± 6.5
BMI (kg/m^2^)	21.5 ± 0.7
PSA (ng/mL)	69.8 ± 10.4
Duration of diseases (years)	2.5 ± 0.6
BPH (*n*)	23
Intraepithelial neoplasia (*n*)	2
Prostatitis (*n*)	4
Prostate cancer (*n*)	43
Hyperlipidemia (*n*)	12
Hypertension (*n*)	15
Diabetes (*n*)	18

BPH: benign prostatic hyperplasia, PSA: prostate specific antigen, BMI: body mass index.

**Table 2:** Comparison of diagnostic efficiency of CEUS, MRI, and the combined application for prostatic cancer.

Groups	*Pathological examination*		Sensitivity (%)	Specificity (%)
	Benign masses	Malignant masses		
*Contrast-enhanced ultrasound*			72.1	79.3
Benign masses	23	12		
Malignant masses	6	31		

*MRI*			74.4	82.8
Benign masses	24	11		
Malignant masses	5	32		

*Contrast-enhanced ultrasound plus MRI*			90.7	89.7
Benign masses	26	4		
Malignant masses	3	39		

**Table 3:** Comparison of ROC results of CEUS, MRI, and the combined application for prostatic cancer.

Groups	AUC	Se	95%CI
Contrast-enhanced ultrasound	0.608	0.049	0.518∼0.813
MRI	0.667	0.042	0.507∼0.798
Contrast-enhanced ultrasound plus MRI	0.785	0.037	0.642∼0.875

**Table 4:** Comparison of diagnostic efficiency of CEUS combined with MRI among different levels of PSA.

CEUS combined with MRI	4 ng/mL < PSA ≤ 10 ng/mL	10 ng/mL < PSA ≤ 20 ng/mL	PSA > 20 ng/mL
Sensitivity	100% (2/2)	81.8% (9/11)	100% (20/20)
Specificity	78.3% (18/23)	60.0% (6/10)	66.7% (4/6)

## Data Availability

The experimental data used to support the findings of this study are available from the corresponding author upon request.
